# Dynamic Evaluation of Intensive Land Use Based on Objective Empowerment by Entropy Method and Neural Network Algorithm

This article has been retracted.

**DOI:** 10.1155/2022/2429826

**Published:** 2022-08-21

**Authors:** Ting Yang, Hanlie Cheng, Hailian Zhao, David Cadasse

**Affiliations:** ^1^School of Public Administration, Chongqing Technology and Business University, Chongqing 400076, China; ^2^School of Energy Resource, China University of Geosciences (Beijing), Beijing 434000, China; ^3^COSL-EXPRO Testing Services (Tianjin) Co., Ltd., Tianjin 300457, China; ^4^School of Soil and Water Conservation, Beijing Forestry University, Beijing 100083, China; ^5^The King's School, BP1560, Bujumbura, Burundi

## Abstract

In the past, the extreme value standardization of indicators, the traditional weighting method, and the multifactor comprehensive model of land intensive use inevitably linearly correlate the evaluation indicators with the evaluation objects, ignoring the direction differences of different indicators in different intervals. At the same time, these methods are also difficult to meet the change of evaluation index weight value with land use type, and cannot adapt to the actual situation of land use environment level and dynamic change. Considering the objectivity of nonlinear correlation moderate index and weight assignment, based on the standardization of quadratic function index and entropy assignment, this paper studies the intensive and dynamic use of land in development zones by different regions to improve the realistic fit of the evaluation model. The results show that the overall level of land intensive use in Chongqing center district and western Chongqing is better than that in northeast Chongqing and southeast Chongqing, roughly showing the state of “high in west and low in east.”

## 1. Introduction

The more China promotes high-quality economic and social development and promotes ecological civilization construction, the more it needs to economize and make intensive use of every inch of nonrenewable land. Facing the dual pressure of protecting resources and ensuring development, the economical and intensive use of land has become an inevitable choice to change the way of land use, optimize resource allocation, expand new drivers of economic development, and make use of stock space [1–4]. At present, scholars and experts have carried out a lot of studies on land intensive use evaluation, internal coordination analysis, influencing factors research, evaluation index system construction, etc. [5–10]. Land intensive utilization evaluation method concentrates multifactor comprehensive evaluation method, the neural network algorithm, principal component analysis (PCA), the fuzzy hierarchy comprehensive evaluation method, etc. The neural network algorithm by selecting the evaluation index factor and factor of unit works is quantified by the appropriate model, calculation and merge, so as to realize the evaluation target; this is the most commonly used method. For example, standard deviation standardization method, ratio standardization method, range standardization method, etc, are common in calculation, while moderate index is often segmented, and positive index calculation method is adopted when the value is less than the ideal value, without fully considering the nonlinear relationship between evaluation index and evaluation result [11–17]. While positive correlation and negative correlation indicators in the evaluation of land intensive utilization is the most common, but the land use structure indicators such as plot ratio and building density, as well as appropriate population density, ratio and other indicators, as well as the commonly used dimensionless index method, cannot eliminate the difference in characteristics, and are prone to overestimate some information loss caused by the level of intensity [18–22]. Based on the quadratic function indicator standardization evaluation index/evaluation results of both nonlinear relationship, it selects the index weight objective empowerment; confirm dynamic entropy weight-driven value analysis was used to explore the change of land intensive use in different time span; entropy index between different sizes directly reflects the degree of target state changes; the overall difference between limit and driving factors avoids the influence of human factors of subjective weighting methods such as Delphi method, analytic hierarchy process, and factor pair comparison method, improves the accuracy and effectiveness of calculation results, and improves the realistic goodness of fit of the evaluation model.

## 2. Research Methods and Data Sources

### 2.1. Research Methods

#### 2.1.1. Standardization of Quadratic Function Indexes

The theoretical basis for the standardization of quadratic function indexes is the law of diminishing marginal utility. The land users in the study area are set as consumers, the standardized value of indicators is set as utility, and the actual value of indicators is set as consumption units. The process of intensive land users is the process of utility satisfaction of land users, and the behavior associated with appropriate indicators according to the law of diminishing marginal utility.

There are *n* quantitative evaluation indexes *X*1, *X*2,…, *Xn*, and *m* samples constitute the index data matrix *P*={*Xij*}(*i*=1,2,…, *m*; *j*=1,2,…, *n*); *Xij* represents the value of the *j* item evaluation index of the ith sample. The current value of the *j* index is *Xj*. The ideal value of evaluation index Xj is X0. Weight is *Wj*; The standardized value is *Yj*, and the standardized formula of the quadratic function index is *Yj*=*aXj*2+*bXj*.

When the actual value of the evaluation index *Xj* reaches the ideal state *X*0, it should be 1 after standardized treatment, and the evaluation value of the quadratic function index formed after standardization is between [0,1]. The ideal value is *X*0. According to the function fixed point value [*X*0,1] and [0,0], parameters a and *b* in the model can be calculated:

(1) $$\begin{array}{c} b=\frac{2}{X_{0}},a=\frac{1}{X_{0}}. \end{array}$$

The improved calculation method of combination index standardization method is shown in formulas (1)–(3). A multifactor evaluation model is formed as formula (5), where *J* represents the land intensity score of the study area:

(2) $$\begin{array}{c} \text{positive indicators }Yj=\frac{\left(Xj-X\min\right)}{\left(X\max-Xmin\right)}, \end{array}$$

(3) $$\begin{array}{c} \text{negative indicators }Yj=aXj2+bXj, \end{array}$$

(4) $$\begin{array}{c} \text{appropriate indicators }Yj=\frac{\left(X\max-Xj\right)}{\left(X\max-Xmin\right)}, \end{array}$$

(5) $$\begin{array}{c} J=\sum_{j=1}^{n}\left(W_{i}\times y_{j}\times 100\right). \end{array}$$

Take the derivative of *J* with respect to *Yj* in formula (4), the derivative of *Yj* with respect to Xj in formulas( 1) and (3), *J*' = 100×*Wj*. Positive indicators: *Yj*' = 1/(Xmax－Xmin). Negative indicators:Yj' = －1/(Xmax－Xmin); it can be seen that the land intensity score *J* is linearly correlated with the standardized index Yj; appropriate indicators Yj in (5) is: J' = 100×*Wj* (2*aXj* + *b*); it can be seen that the land intensity score *J* is linearly correlated with the standardized index *Yj*.

#### 2.1.2. Entropy Value Method

In comprehensive evaluation, it is generally believed that the index weight value determined by entropy method is more objective and more reliable than the subjective weight method such as Delphi method and analytic hierarchy process. Entropy method is based on the information entropy theory. According to the difference of the information order degree contained in each evaluation index, the higher the order degree of a system is, the greater the information entropy is and the smaller its utility value is. Different entropy values between indicators are generally applicable for weight determination in time series evaluation. To calculate the index entropy *e*_*j*_, the formula is as follows:

(6) $$\begin{array}{c} e_{j}=-\frac{1}{\text{In}m}\sum_{i-1}^{m}P_{ij}\times \text{In}P_{ij}. \end{array}$$

Among them, *P*_*ij*_ is the contribution degree of a single indicator. The weight *Wj* is calculated by using the entropy value obtained, and the calculation formula is as follows:

(7) $$\begin{array}{c} W_{j}=\frac{gi}{\sum_{j-1}^{n}gi}. \end{array}$$

*Wj* is the weight of the *j* index, and *gi* is the difference coefficient of the *j* index.

### 2.2. The Data Source

The data were mainly obtained from Chongqing Land use status change survey data, statistical yearbook from 2014 to 2018, land use and enterprise survey data of development zone, dynamic monitoring and supervision system data of land market, Urban and Rural Development Commission, natural Resources Bureau, etc.

## 3. The Study Area

As an important area of regional economic development, the development zone is the scientific and technological innovation base of industrial upgrading and regional development and also an important growth point of the sustainable development of urban economy. As of 2018, Chongqing has eight national development zones and forty-one provincial-level development zones, including Xiyong Comprehensive Bonded Zone, Lianglu-Cuntan Free Trade Port Area, Chongqing Economic and Technological Development Zone, and Chongqing High-Tech industry development Zone. There are forty-nine development zones in total which have greatly promoted regional economic development. Based on the characteristic support development zone system of Chongqing center district, western Chongqing, northeast Chongqing, and southeast Chongqing as an example, this paper evaluated the dynamic situation of land intensive use from 2013 to 2017 by combining the quadratic function index standardization and entropy method weighting method. By the end of 2017, the Chongqing development zone covers an area of 665.97 square kilometers, with a land development rate of 71.23%, a total resident population of 2.0741 million, a total investment in industrial fixed assets of 1.149247 billion, and a total industrial tax revenue of 50.902 billion.

## 4. Result Analysis

### 4.1. Establishment of the Evaluation Index System

In this paper, a total of ten indicators *C*1 − 1/*C*10 − 1) are selected as the evaluation indicators of the Industrial-led Development Zone, and seven indicators *C*1 − 2/*C*10 − 2 are selected as the evaluation indicators of the City-industry integration development zone, in which the idle rate of land *C*10 − 1/*C*10 − 2 is a negative indicator, and the building density *C*5 − 1/*C*5 − 2 and population density (C9-2) are appropriate indicators(Table 1). After the standardization of the evaluation index by the quadratic function, the ideal value of the evaluation index of building density in Chongqing center district at the end of 2017 is 56.83%, and the quadratic function value *Y* = 2.149. The ideal value of the evaluation index of population density is 383.66 people/hectare, and the quadratic function value *Y* = 1.422. The other evaluation indexes are all positive indicators.

### 4.2. Weight Analysis of Evaluation Indicators

The rationality of index weight directly affects the order of pros and cons of evaluation objects, thus greatly affecting the accuracy of comprehensive evaluation. The weight values of dynamic indicators of the industrial-led development zone are determined according to the entropy method, as shown in Table 2. The entropy weight of the city-industry integration development zone is WC1-2 = 0.122, WC2-2 = 0.124, WC4-2 = 0.121, WC5-2 = 0.125, WC8-2 = 0.143, WC9-2 = 0.121, and WC10-2 = 0.244.

### 4.3. Dynamic Comparative Analysis of Land Use Status

According to the analysis of the current situation values in different years, the land supply rate of development zones in Chongqing center district (A), western Chongqing (B), northeast Chongqing (C), and southeast Chongqing (D) was basically flat, which were all at Chongqing center district high level, respectively, 91.60%, 89.33%, 86.23% and 89.51%. The area with the best land supply is Chongqing center district, and the area with the greatest supply potential is northeast Chongqing. The land construction rate, respectively, is 80.53%, 75.43%, 71.73%, and 67.40%. Chongqing center district has superior location conditions, and the soft and hard environmental conditions for industrial development are better. The land construction rate is the highest. Compared with the land supply rate of 84.26%, 89.71%, 87.52%, and 64.4% in 2013, and the land construction rate of 83.57%, 97.09%, 87.83%, and 82.72% in 2013, the land development rate in Chongqing center district, western Chongqing, and northeast Chongqing showed an overall trend of first decreasing and then increasing. The area in southeast Chongqing showed a trend of first rise and then decline, and the land construction rate showed a trend of saturation decline as a whole, as shown in Figure 1.

In terms of land use structure, intensity and benefit, the industrial land use rate in western Chongqing is higher than that in other three areas, and its dynamic change reaches the highest value of 76.39% in four years. Except for southeast Chongqing, the building density, comprehensive floor area ratio of industrial land, building coefficient of industrial land, and fixed asset input intensity of industrial land in the other three regions all showed an upward trend. The average tax revenue of industrial land in western Chongqing, northeast Chongqing, and southeast Chongqing was basically stable. By the end of 2017, there are 0.0.9% and 0.7% of idle land in Chongqing center district and southeast Chongqing, and the rate of idle land was relatively low. There is no idle land in western Chongqing and northeast Chongqing, and the land management performance is good. For newly built has not yet been put into production, the stable industrial land scale is larger; Chongqing center district has 0.09% idle land, leading to the both of industrial land tax with the year dropped substantially.

### 4.4. A Case Study on Comprehensive Evaluation of Land Use Intensity

According to the weight value of each evaluation index, the status value of the index ranked fifth was used as the ideal value of the corresponding index; after the standardization of indicators, the comprehensive score of land intensity was calculated. It can be divided into four grades: extensive utilization (<60), preliminary intensive utilization (60–70), basic intensive utilization (70–80), and highly intensive utilization (80–100).

On the whole, the intensity score of 49 development zones in Chongqing presents a state of “high in the west and low in the east.” Chongqing center district is the political, economic, cultural, modern service center, and population agglomeration area of the whole city, and the development environment of high-tech industry is good. The second area is western Chongqing. As an important manufacturing base of the whole city, western Chongqing is an important area to gather new industries and population. The overall level of land intensive use in Chongqing center district and western Chongqing is better than that in northeast Chongqing and southeast Chongqing. 92% of the development zones of type I highly intensive utilization grade are distributed in Chongqing center district and western Chongqing. Only three development zones in the whole city have the intensity score exceeding 90 points, including Chongqing Gangcheng Industrial Park in Chongqing center district 92.33 points, Chongqing Tongxing Industrial Park in Chongqing center district 90.70 points, and Chongqing Fuling Industrial Park in western Chongqing 92.38 points. There are 20 development zones of basic intensive utilization grade II, which are distributed in all four zones. Due to the limitation of terrain conditions in northeast Chongqing and southeast Chongqing, the land area of development zone is relatively small and the building coefficient of industrial land is relatively high, due to the large proportion of transportation land, public management land, and public service land in the development zone of northeast Chongqing; the realization rate of paid land use in the development zone is reduced to a certain extent, and the marketization degree of land supply is the lowest. The lowest score of intensity in northeast Chongqing is 50.83 in Chongqing Jiangjin Comprehensive Bonded Tax Zone and 56.19 in Chongqing Fengjie Industrial Park in western Chongqing, both of which belong to type IV extensive utilization grade. The development zones with the grade III of preliminary intensive utilization include Changshou Economic and Technological Development Zone with 67.04 points, Chongqing Chengkou Industrial Park with 61.40 points, and Chongqing Pengshui Industrial Park with 69.15 points.

Compared with the four regions in the time series, the Central District of Chongqing has the highest land intensity in the past four years, and the land intensity in the Central District of Chongqing has decreased year by year. However, at a high level, the degree of land intensity in the western part of Chongqing is increasing year by year. The central area of Chongqing and the western part of Chongqing both maintained above 80 points, and the northeast of Chongqing showed a trend of first decreasing and then slightly increasing, reflecting the basic intensive utilization level. Southeast Chongqing showed a trend of first slight increase and then strong decrease, as shown in Figure 2.

## 5. Conclusion

From the perspective of the change of the dynamic evaluation result data and the comprehensive function development of the development zone, in recent years, the Chongqing development zone are higher than the average level of the national development zones in the same year. The space for improving land use structure and land use intensity is gradually shrinking, and the overall level of intensity is relatively high. The development zone has been transformed from a single industrial park to an urban comprehensive functional zone, the land use structure has been further rationalized, and the supply of infrastructure facilities and public service land has increased. Compared with the changes over the years and the national level, the short board of land intensive use in Chongqing Development Zone lies in the low land use efficiency. Industrial land is below the national average national level development zone in the same year tax, and the comprehensive benefits of play is not enough.

The Chongqing development zone should be through the industry upgrading and transfer, improve the level and quality of land output per unit area, and reduce the consumption of social economic development on the land. The extensive road of development by relying on land expansion can no longer continue. The development mode of land use should be changed to further release the longitudinal and vertical space of internal land use. Tap the potential and invigorate the stock, and improve the postsupply supervision mechanism, to achieve the connotative intensive and sustainable development.

## Figures and Tables

**Figure 1:** Statistical chart of the current value of land intensive and economical use in the development zone.

**Figure 2:** Dynamic change of land use intensity score from 2013 to 2017.

**Table 1:** Evaluation index system of intensive utilization in the development zone.

The target layer A	Rule layer B	Index layer C	Index meaning
Land use status A1	Degree of land use B1	Land supply rate *C*1 − 1/*C*1 − 2	Refers to the ratio of the area of state-owned construction land already supplied to the area of land already supplied
		Land construction rate *C*2 − 1/*C*2 − 2	Refers to the ratio of built-up urban construction land area to state-owned construction land area
	Land use structure B2	Industrial land ratio C3-1	Refers to the percentage of industrial, mining and storage land area within the scope of built-up urban construction land and built-up urban construction land area
	Land use intensity B3	Combined volume ratio *C*4 − 1/*C*5 − 2	Refers to the ratio of the total built-up area on the built-up urban construction land to the built-up urban construction land area
		Building density *C*5 − 1/*C*5 − 2	Refers to the ratio of the total area of building basement within the completed urban construction land to the completed urban construction land area
		Comprehensive plot ratio of industrial land C6-1	Refers to the ratio of total built-up area of industrial land to industrial land area
		Building coefficient of industrial land C7-1	Refers to the percentage of built-up area of industrial land to industrial land
Land use efficiency A2	Industrial land input output benefit B4	Fixed asset input intensity of industrial land C8-1/Comprehensively equalize taxation C8-2	Refers to the ratio of accumulated fixed asset investment of industrial (logistics) enterprises within the scope of land used for urban construction to the area of land used for industrial, mining, and storage/refers to the ratio of total tax revenue of secondary and tertiary industries within the scope of land used for urban construction to the area of land used for urban construction
		Average tax on industrial land C9-1/The population density C9-2	Refers to the ratio of total tax revenue of industrial (logistics) enterprises within the scope of completed urban construction land to the area of industrial, mining and storage land/refers to the ratio of permanent resident population within the scope of evaluation to the area of completed urban construction land
Land management performance A3	Land use regulatory performance B5	Idle rate of land *C*10 − 1/*C*10 − 2	Refers to the ratio of idle land area to the development zone area

**Table 2:** Index weights of the time series.

The target layer	Land use status							Land use efficiency		Land management performance
Index layer	C1	C2	C3	C4	C5	C6	C7	C8	C9	C10
2013	0.559							0.191		0.250
	0.053	0.119	0.055	0.118	0.102	0.060	0.052	0.071	0.120	0.250
2015	0.550							0.168		0.282
	0.073	0.061	0.083	0.106	0.082	0.063	0.081	0.070	0.099	0.282
2017	0.739							0.202		0.059
	0.066	0.078	0.095	0.142	0.076	0.088	0.194	0.139	0.063	0.059

## Data Availability

The figures and tables used to support the findings of this study are included in the article.
